# Spironolactone Inhibits Cardiomyocyte Hypertrophy by Regulating the Ca^2+^/Calcineurin/p-NFATc3 Pathway

**DOI:** 10.1155/2021/3843830

**Published:** 2021-12-16

**Authors:** Xin Wang, Wenting Zhang, Jingtao Na, Yanping Huo, Yacheng Wang, Ketong Liu

**Affiliations:** ^1^Department of Cardiovascular Medicine, The Third Affiliated Hospital of Qiqihar Medical University, Qiqihar 161000, China; ^2^Department of Clinical Pharmacy, The Third Affiliated Hospital of Qiqihar Medical University, Qiqihar 161000, China; ^3^The Ultrasound Department, The Second Hospital of Qiqihar, Qiqihar 161000, China

## Abstract

This study aimed to investigate the protective effect and molecular mechanism of spironolactone in isoproterenol-induced cardiomyocyte hypertrophy. In this study, primary cardiomyocytes were extracted from the heart of neonatal rats. After stable culture, they were processed with isoproterenol alone or isoproterenol (10 *μ*M) combined with different doses (low dose of 10 *μ*M and high dose of 50 *μ*M), and the cellular activity was determined by MTT experiment. The volume of cells was measured with an inverted microscope and CIAS-1000 cell image analysis system. The mRNA expression levels of ANP and BNP in cells were explored by RT-qPCR. The levels of ANP and BNP proteins and NFATc3 phosphorylation in the nucleus were detected by western blot. The extracellular Ca2^+^ concentration and CaN activity were measured by colorimetry with the kit. Isoproterenol significantly enlarged the volume of cardiomyocytes (*p* < 0.001), upregulated mRNA and expression levels of ANP and BNP proteins (*p* < 0.001), increased extracellular Ca^2+^ concentration and CaN activity (*p* < 0.001), and upregulated NFATc3 phosphorylation in the nucleus (*p* < 0.001). The volume of cells treated with isoproterenol combined with different doses of spironolactone significantly decreased compared with those treated with isoproterenol alone (*p* < 0.001). mRNA and expression levels of ANP and BNP proteins downregulated significantly (*p* < 0.001). The extracellular Ca^2+^ (*p* < 0.01) concentration and CaN activity (*p* < 0.001) decreased significantly, and NFATc3 phosphorylation in the nucleus downregulated significantly (*p* < 0.001). There was no significant difference in cell volume (*p*=0.999), ANP and BNP mRNA (*p*=0.695), expression levels of proteins, CaN activity (0.154), and NFATc3 phosphorylation in the nucleus between the cells treated with isoproterenol combined with high-dose spironolactone and those in the control group. In conclusion, spironolactone can reverse isoproterenol-induced cardiomyocyte hypertrophy by inhibiting the Ca^2+^/CaN/NFATc3 pathway.

## 1. Introduction

The main inducement of cardiomyopathy-induced hypertrophy is long-term abnormal hemodynamics caused by hypertension, myocardial infarction, and other factors [1, 2], in which myocardial remodeling is the key pathological stage. It is the dynamic pathological process of abnormal biological characteristics of cardiomyocytes and their imbalance with noncardiomyocytes under stress [3, 4]. Long-term pathophysiological studies have shown that abnormal metabolism and proliferation of cardiomyocytes, participation of noncoding RNA, immune response, transcriptional regulation, and epigenetic modification all play important roles in cardiomyocyte remodeling [5, 6]. Besides, some cytokines (proinflammatory factors, coagulation factors, etc.) and proteases (collagen, calcineurin, etc.) activate or inhibit myocardial remodeling-related signaling pathways at the subcellular level or can become clinically effective targets for molecular intervention [1, 7, 8].

CaN is a kind of protein phosphatase regulated by Ca^2+^/calmodulin, which regulates the expression of intranuclear genes (ANP, BNP, etc.) by translocation of an activated *T* nuclear factor (NFAT3) into the nucleus [9–13]. The latest research shows that the CaN-NFAT pathway in rats was inhibited, where Ca^2+^/calmodulin-dependent protein kinases *β*-*γ*-related genes have been knocked out. It is not easy to form pathological myocardial hypertrophy [14, 15]. The molecular mechanism of CaN-NFAT-mediated myocardial remodeling is the significant downregulation of interferon 8 (IFN 8) in the body of cardiac hypertrophy. IFN 8 CaN interacts with NFAT and inhibits NFAT from entering the nucleus to play a regulatory role [16]. To sum up, the Ca^2+^-mediated CaN/NFAT pathway plays a vital part in the occurrence and development of myocardial hypertrophy [13, 17].

Spironolactone, a nonselective salt corticosteroid receptor antagonist, is widely used in the therapy of water and sodium retention [18]. Recent research reports that spironolactone can reduce cardiac preload, ameliorate cardiac pump ability, and improve survival rate in patients with symptomatic heart failure and postmyocardial infarction systolic dysfunction, with obvious prognostic benefits in patients with heart failure [19–21]. However, there is no specific report on the positive therapeutic significance of spironolactone on myocardial hypertrophy and no further exploration of relevant mechanisms. This study aims to explore the effect of spironolactone on myocardial hypertrophy and its mechanism based on isoproterenol-induced cardiomyocyte hypertrophy. This study confirmed that the Ca^2+^/CaN/p-NFATc3 pathway is related to the protective effect of spironolactone and did not confirm that the pathway has a direct effect, which needs further study.

## 2. Method

### 2.1. Extraction of Cardiomyocytes from Primary Neonatal Rats

SD neonatal rats born within 72 h were used (parental rats were purchased from Vital River, License No.: SCXK (Shanghai)). The rat was anesthetized with a small animal anesthesia machine (2% isoflurane, 0.25 L/min) and disinfected with iodophor 3 times after satisfactory anesthesia. After regularly placing the towel, the chest of the rat was cut to expose the heart, which was taken out, with the arteries cutting out, and placed in a precooled PBS buffer (KGB5001, KeyGEN BioTECH, containing a mixture of penicillin, KGY0023). The blood clots around the heart were removed with ophthalmic scissors, and the heart was cut and washed 3 times with the buffer to rinse the remaining blood. 5 ml of trypsin solution (concentration: 0.25%, KGM25200, KeyGEN) was injected into the heart, with the agitating magnetons added to the magnetic stirrer and digesting at 60 rpm, 37°C, for 15 min. After digestion, the supernatant was added with 10 ml trypsin solution and fully mixed, and the agitating magnetons were added to the magnetic stirrer and were digested at 60 rpm, 37°C, for 10 min again. The abovementioned absorption and digestion steps were repeated. After two times of digestion, the solution was passed through a 200-mesh screen, centrifuged at 2000 rpm for 10 min, resuspended with 8 ml DMEM medium (11995073, Gibco, Thermo Fisher) containing 20% fetal bovine serum (FBS, 16140071, Gibco, Thermo Fisher), and inoculated in culture dishes. After 90 min, adherent cells were discarded, and the remaining cells suspended in the medium were inoculated in a new Petri dish at a density of 5 × 10^5^ cells/mL, and cultured in 5% carbon dioxide at 37°C for 24 h. The floating dead cells were removed, and the medium was replaced to prepare for subsequent experiments. All cell extraction procedures were carried out at room temperature.

### 2.2. Cell Culture and Experimental Grouping

After 72 h of stable culture, the extracted cardiomyocytes have further interfered. In order to ensure the activity of cardiomyocytes, all the cells were extracted from rats without cell passage.

Experimental grouping: (1) normal control group (NC); (2) isoproterenol stimulation group (ISO group, isoproterenol concentration 10 M, I5627, Sigma-Aldrich); (3) isoproterenol combined with the low-spironolactone-isoproterenol-stimulation group (low-SPL-ISO group, 10 *μ*M spironolactone, HY-B0561, MCE); and (4) isoproterenol combined with the high-spironolactone-isoproterenol-stimulation group (high-SPL-ISO group, 50 *μ*M spironolactone).

### 2.3. Cell Viability Test

The cell viability (KGA311-KGA312, KeyGEN BioTECH) was detected with MTT colorimetric assay. After 48 h of steady growth, about 1 × 10^4^ cells (about 200 *μ*l) were inoculated into the 96-well plate, divided into groups according to the ignoble method in Section 1.2, and stimulated for 48 h, and 50 *μ*l MTT was added into each well. After incubation at 37°C for 2 h, 150 *μ*l dimethyl sulfoxide (DMSO) was added to dissolve ignoble, and the absorbance value was measured at 480 nm by ELISA (Absorbance 96, Byonoy, Germany). The cell viability compared to the normal control group (%) = (OD measure−OD calibration)/(OD blank−OD calibration) ×100%.

### 2.4. Cell Volume Determination

Four groups of cells were digested and resuspended with a 200 *μ*l DMEM medium. Four fields of view were randomly selected, and the diameter of 20 cells was measured, and the volume was calculated using the cell image analysis system (CIAS-1000, Daheng, Beijing). The cell suspension was injected into the Transwell cell chamber (3422, Corning), and the cell morphology was observed under an inverted microscope with a magnification of 400 times.

### 2.5. Extraction of Nuclear Proteins

Nuclear proteins were extracted with a nuclear extraction kit (KGA826, KeyGEN BioTECH). All operations were performed according to the instructions of the kit. The specific operation steps are as follows: 4 groups of cells were digested and washed twice with PBS (centrifugation at 2000 rpm for 5 min), and 100lL cells (about 1 × 10^7^ cells) were collected. 1 ml ice precooled lysis buffer was added with oscillation and resuspension, with 50 *μ*l reagent A added, followed by oscillation mixing. The cell suspension was placed in an ice-water bath for 20 min, with oscillation 30 s per 5 min. Under the microscope, there should be a large number of free nucleus and a few unlysed cells. The suspension was transferred to a centrifuge tube for centrifugation at 1000 g, 4°C for 3 min. Then, the supernatant was discarded to obtain the nuclear mixture. The nucleus was resuspended with a 500 *μ*l lysis buffer and centrifuged at 1000 g, 4°C, for 3 min; then, the supernatant was discarded. 500 l medium buffer A was added to resuspend the precipitation. The resuspension was placed on 1 ml medium buffer B, centrifuged at 1000 g, 4°C, for 10 min, and relatively pure nuclear precipitation was obtained for subsequent experiments.

### 2.6. Quantitative Real-Time PCR (qRT-PCR)

About 5 × 10^8^ cells in each of four groups were collected, 500 *μ*l TRIzol (R0016, Beyotime) lysate protein nucleic acid complex was added, and 100 *μ*l chloroform was mixed to extract RNA. After centrifugation at 12000 RPM, 4°C, for 10 min, the upper colorless aqueous phase was collected, 200 *μ*l isopropanol was added to precipitate RNA, and 75% of the cells were washed. The extracted RNA was retrotranscribed into a cDNA template with a reverse transcription reagent (RR037Q, Takara). Then, a real-time fluorescent quantitative polymerase chain reaction (Applied Biosystems, ABI 7500) was conducted with TB Green qPCR reagent (RR82LR, Takara). The Ct value of genes to be examined was calibrated using the Ct value of the internal reference gene GAPDH, and the amplification multiple of genes relative to the internal reference genes was calculated according to the 2^−∆∆Ct^ formula. Amplification conditions: the first stage was kept at 95°C for 30 s; the second stage was 95°C for 5 s and 60°C for 30 s, for 40 cycles; and the third stage was maintained at 95°C for 15 s, 60°C for 60 s, and 95°C for 15 s.

#### 2.6.1. Primer Sequences

ANP : F 5′-GGCTCCTTCTCCATCACCAA-3′, *R* 5′-TGTTATCTTCGGTACCG-3';

BNP : F 5′-GATCAAGCTTATGGAT-CCCCAGACAGCACCTTCC-3′, R5′-GATCGAATTCACCGTGGAA-ATTTTGTGCTCAA-3'; and

GAPDH: F 5′-TGATGCTGGTGCTGAGTATG-TCGT-3′, *R* 5'-TCTCGTGGTTCACACCCATCACAA-3'.

### 2.7. Western Blot

About 5 × 10^8^ cells in each of four groups were collected, and 1 ml RIPA protein lysate (KGP704, Kai-Bio) containing 1% protease inhibitor and phosphatase inhibitor (78445, Thermo Fisher Scientific) was added to extract the total protein. The protein concentration was determined using the BCA protein assay kit (P0006, Beyotime), which was diluted to 4 *μ*g/*μ*l with RIPA buffer lysate. SDS-PAGE protein loading buffer (P0015, Beyotime) was added and denaturated at 100°C for 5 min to obtain protein samples. After 50 g of total protein was separated by SDS-PAGE according to molecular weight, the target protein was transferred to the PVDF membrane (T2234, Thermo Fisher Scientific). The membrane was sealed with a blocking buffer (P0252, Beyotime) for 1 h at room temperature, and anti-BNP (1 : 2000, AB243440, ABCAM), P-NFATC3 (1 : 1000, AB59204, ABCAM), T-NFATC3 (1 : 3000, AB93628, ABCAM), *β*-actin (1 : 8000, AB179467, ABCAM), and anti-GAPDH (1 : 5000, AB181602) were added. Abcam antibodies were incubated at 4°C overnight. HRP-labeled sheep anti-rabbit (Abcam, AB205718, 1 : 10,000) secondary antibody was added after washing 3 times with TBST and incubated at room temperature for 2 h. After washing 3 times with TBST, ECL luminescent solution (P10300, New Cell & Molecular Biotech, Suzhou) was adopted for development in the chemiluminescence system (Millipore Corporation, Billerica), and Image *J* (NIH, Bethesda) was adopted for grayscale analysis of the strips.

### 2.8. Determination of Ca^2+^ Concentration

Ca^2+^ concentration in the cell medium was determined by the colorimetric method with a Ca^2+^ concentration determination kit (K380-250, Shanghai Yubo Biotechnology). 10 *μ*l medium for each of the four groups was collected; 90 *μ*l chromotropic solution was added and diluted with 60 *μ*l buffer solution. The cells were incubated for 15 min in the dark at room temperature, and the absorbance value was detected at 550 nm wavelength by ELISA (Absorbance 96, Byonoy, Germany).

### 2.9. Detection of Calcineurin Phosphatase Activity

According to the product description, the calcineurin phosphatase activity in cells was detected by the colorimetric method using the kit (ab139461, Abcam). The culture medium of the four groups of cells was collected for 20 *μ*l in each, with 380 *μ*l enzyme luminescent substrate added. After incubation at room temperature for 30 min, the absorptivity was detected at 660 nm wavelength by ELISA (Absorbance 96, Byonoy, Germany).

### 2.10. Statistical Methods

All data in this study were numerical variables, and a postverb *t*-test was conducted with univariate analysis of variance and Turkey's multiple-verb test based on SPSS 19.0 software. Data were expressed as *x* ± *s*, and *p* < 0.05 was defined as the difference that was statistically significant (^*∗*^*p* < 0.05, ^*∗∗*^*p* < 0.01, ^*∗∗∗*^*p* < 0.001, and NS: no significance).

## 3. Results

### 3.1. Effects of Different Stimuli on Cell Viability

In order to explore whether each stimulus had an effect on cell viability and whether the status of cells was at a uniform level, the cell viability of each group relative to the normal control group was evaluated with the MTT method. It turns out that the treatment of 10 *μ*m isoproterenol alone (ISO group) or isoproterenol combined with 10 *μ*m and 50 *μ*m spironolactone (low-SPL-ISO group and high-SPL-ISO group) had no effect on cell viability (*F* = 1.148, *p*=0.360), with no significant difference, as shown in Figure 1.

### 3.2. Effects of Different Treatment Factors on the Volume of Cardiomyocytes

In order to intuitively explore the protective effect of spironolactone on isoproterenol-induced cardiomyocyte hypertrophy, an inverted microscope was utilized to randomly select 4 fields of vision with the cell image analysis system to measure the diameter and calculate the volume of 20 cells. The results showed that the volume of cells in each group was significantly different under different treatment factors (*F* = 64.47, *p* < 0.001), the isoproterenol-treated cardiomyocytes were significantly larger than those in the blank control group (*q* = 16.68, *p* < 0.001), the volume of cardiomyocytes treated with low- and high-concentration spironolactone was significantly smaller than that in the isoproterenol-treated group alone (*q*_1_ = 7.31, *q*_2_ = 16.45, all *p* < 0.001), and high-concentration spironolactone effect was more obvious. These results suggest that spironolactone can significantly reverse isoproterenol-induced cardiomyocyte hypertrophy in a dose-dependent manner, as shown in Figure 2.

### 3.3. mRNA and Expression Levels of ANP and BNP Proteins in Cardiomyocytes of Each Group

In order to further verify the protective effect of spironolactone on isoproterenol-induced cardiomyocyte hypertrophy at the molecular marker level, this study explored the expression levels of myocardial injury markers ANP and BNP at the mRNA and protein levels. The results showed that there were significant differences in the mRNA expression of ANP and BNP in cardiomyocytes of different treatment factors (*F*_ANP_ = 95.14, *F*_BNP_ = 195.4, all *p* < 0.001), in which the expression of ANP (*q* = 20.67, *p* < 0.001) and BNP (*q* = 29.85, *p* < 0.001) in cardiomyocytes treated with isoproterenol was significantly higher than that in the normal control group. Low and high concentrations of spironolactone could significantly reduce the high mRNA expression level of ANP (*q*_1_ = 8.07, *q*_2_ = 19.12, all *p* < 0.001) and BNP *(q*_1_ = 17.62, *q*_2_ = 28.29, all *p* < 0.001) in cardiomyocytes induced by isoproterenol. There was no significant difference in the mRNA level of ANP (*q* = 1.56, *p*=0.695) and BNP (*q* = 0.57, *p*=0.978) in myocardial cells treated with high-concentration spironolactone compared with the blank control group, as shown in Figure 3(a). The expressions of ANP and BNP in each group were consistent with mRNA, and spironolactone could dose-dependently decrease the levels of ANP and BNP in isoproterenol-treated cardiomyocytes, as shown in Figure 3(b). All these results suggest that spironolactone can dose-dependently reverse the high levels of ANP and BNP in cardiomyocytes induced by isoproterenol.

### 3.4. Extracellular Ca^2+^ Concentration of Cardiomyocytes in Groups

Extracellular Ca^2+^ concentration of cardiomyocytes was detected in order to investigate the mechanism of spironolactone protecting isoproterenol-induced cardiomyocyte hypertrophy. Also, the results showed that the extracellular Ca^2+^ concentration of each group was significantly different (*F* = 38.70, *p* < 0.001), in which isoproterenol significantly increased the extracellular Ca^2+^ concentration of cardiomyocytes (*q* = 14.63, *p q* = 0.001), and low and high concentrations of spironolactone decreased extracellular Ca^2+^ concentration (*q*_1_ = 5.25, *p*_1_ _=_ 0.009; *q*_2_ _=_ 9.50, *p*_2_ < 0.001) in a dose-dependent manner. Changes in Ca^2+^ concentration suggested that the protective effects of spironolactone on cardiomyocytes may be related to Ca^2+^-related pathways, as shown in Figure 4.

### 3.5. CaN Activities of Calcineurin in Cardiomyocytes of Each Group

CaN, as key proteases that activate downstream Ca^2+^ pathways, can promote cardiomyocyte hypertrophy. In this study, CaN activity was detected by ELISA, showing a significant difference in CaN activity in each group under the intervention of different stimulants (*F* = 18.16, *p* < 0.001), in which isoproterenol significantly enhanced the CaN activity in cardiomyocytes (*q* = 9.49, *p* < 0.001). A low concentration of spironolactone significantly attenuated isoproterenol-induced CaN high activity (*q* = 6.75, *p*=0.001), and the effect of high-concentration spironolactone was obvious (*q* = 8.43, *p* < 0.001). CaN activity in cardiomyocytes treated with low and high concentrations was not different from that in the normal control group (*q*_1_ = 2.74, *p*_1_ _=_ 0.254; *q*_2_ _=_ 0.876, *p*_2_ < 0.001). These results suggested that spironolactone can protect cardiomyocytes from isoproterenol damage by inhibiting CaN activity, as shown in Figure 5.

### 3.6. NFATc3 Phosphorylation in the Nucleus of Cardiomyocytes of Each Group

NFATc3 is a key molecule downstream of the Ca^2+^/CaN pathway. This study investigated NFATc3 phosphorylation in the nucleus of each group with western blot. The results showed that NFATc3 phosphorylation was significantly upregulated in isoproterenol-stimulated cardiomyocytes, which was reversed under spironolactone stimulation. Low and high concentrations of spironolactone could significantly downregulate NFATc3 phosphorylation in cardiomyocytes in a dose-dependent manner, as shown in Figure 6. These results showed that Ca^2+^CaN/p-NFATc3 may be a potential signaling pathway for spironolactone to reverse cardiomyocyte hypertrophy.

## 4. Discussion

Based on primary cardiomyocytes, this study explored the protective effect of spironolactone on cardiomyocyte hypertrophy and its molecular mechanism. The results showed that spironolactone can significantly reduce the volume enlargement of isoproterenol-induced cardiomyocytes and downregulate the expression of myocardial injury markers ANP and BNP, suggesting that spironolactone can protect cardiomyocytes from isoproterenol damage in a dose-dependent manner. Further molecular mechanism studies have shown that spironolactone participates in the regulation of cardiomyocyte development by reducing CaN activity and NFATc3 translocation phosphorylation in order to protect cardiomyocytes. A study of the role of spironolactone in cardiomyocyte hypertrophy was presented, and it first reported that spironolactone inhibits cardiomyocyte hypertrophy by regulating Ca^2+^/CaN/NFATc3 pathways.

The heart must pump blood to provide oxygen and nutrition to the body, which consumes a lot of energy, so the heart is equipped with multiple complex biological systems to meet the systemic needs [22]. Normal physiological hypertrophy of the myocardium is associated with angiogenesis and metabolic plasticity and maintenance of cardiac homeostasis during childhood growth, pregnancy, and exercise. Pathological myocardial hypertrophy is caused by long-term abnormal hemodynamic pressure and other factors associated with fibrosis, capillary sparsity, increased production of proinflammatory factors, and cellular dysfunction (impaired signal transduction) [1, 23, 24]. *β*-receptor agonist isoproterenol can excite the myocardial *β*1-receptor, enhance myocardial contractility, accelerate heart rate, increase cardiac output and myocardial oxygen consumption, and increase myocardial load, leading to abnormal cardiomyocytes [25, 26]. In this study, isoproterenol was used for model cardiomyocyte hypertrophy, which is stable and reliable. To investigate whether modeling doses of isoproterenol and low and high doses of spironolactone have an effect on cardiomyocyte viability, MTT experiments were carried out to measure cell viability, showing that the level of cell status was the same with the intervention of 10 *μ*m isoproterenol and 10 *μ*m and 50 *μ*m spironolactone compared between each group.

In recent years, the role of potassium-preserving diuretic spironolactone has been studied in the cardiovascular field [18], especially in the correlation between myocardial remodeling and left ventricular ejection fraction [19–21]. Additionally, spironolactone combined with other drugs can significantly improve various cardiovascular diseases. For example, perindopril combined with spironolactone can significantly inhibit cardiovascular remodeling. High-dose spironolactone combined with glucocorticoid can effectively improve chronic heart failure. These studies suggest that spironolactone has some clinical significance in the treatment of cardiovascular disease [27, 28]. In this study, we found that treatment with spironolactone alone can significantly reduce the volume of cardiomyocytes, inhibit myocardial hypertrophy at the cellular level, and reduce the high level of related markers caused by isoproterenol intervention at the same time. When the myocardium is damaged, ANP and BNP compensatory increases; therefore, myocardial injury and its degree were evaluated with the two clinically stable and sensitive markers [29–32]. In isoproterenol-induced cardiomyocytes, ANP and BNP were upregulated at both mRNA and protein levels, suggesting that isoproterenol can stabilize myocyte injury, and the modified model method is stable and reliable. After a combination of low and high doses of spironolactone, ANP and BNP levels in damaged cardiomyocytes were significantly downregulated, suggesting that spironolactone can effectively protect cardiomyocytes from isoproterenol injury at low levels.

For further investigation of the potential molecular mechanism of spironolactone protecting cardiomyocytes, this study started from the Ca^2+^-related pathway. According to the relevant literature, the Ca^2+^ level significantly upregulated CaN activity, which made NFATc3 into the nucleus to release related proteins from cardiomyocytes, promoting cardiomyocyte injury and then increasing the level of ANP and BNP in cells. During this study, isoproterenol significantly increased the Ca^2+^ level in the cytoplasm, increased CaN activity, and then, upregulated NFATc3 phosphorylation in the nucleus. The combination of low- and high-dose spironolactone significantly inhibited CaN activity and downregulated NFATc3 phosphorylation in the nucleus. Previous data showed that CaN dephosphorylates NFATc3 into the nucleus generating a series of subsequent effects during myocardial injury. In this study, no differences in the levels of NFATc3 proteins were detected in each group. However, there were significant differences in phosphorylation levels between groups, suggesting that NFATc3 nuclear phosphorylation may be a key link in myocardial injury and spironolactone can significantly downregulate high activation of isoproterenol-induced Ca^2+^CaN/p-NFATc3, which may be the mechanism by which spironolactone produces cardiomyocyte protection at a subcellular level.

## 5. Conclusions

This study has the following shortcomings to be further studied. First, this study was based on the cell level, which cannot successfully simulate the complex situation of the body system, so the follow-up study should deeply explore the animal level and then use clinical experiments to clarify the protective effect of spironolactone on myocardial protection. Second, this study focused on the NFATc3 phosphorylation and did not detect the difference in the content of NFATc3 protein, which is inconsistent with the existing literature, so the mechanism of the subcellular level needs to be further explored. Finally, this study confirmed that the Ca^2+^/CaN/p-NFATc3 pathway is related to the protective effect of spironolactone and did not confirm that the pathway has a direct effect, which needs further study.

In conclusion, spironolactone can downregulate NFATc3 phosphorylation in the nucleus of cardiomyocytes by reducing extracellular Ca^2+^ concentration and weakening CaN activity, thus protecting cardiomyocytes.

## Figures and Tables

**Figure 1:** Effects of different stimuli on cell viability.

**Figure 2:** Effects of different treatment factors on the volume of cardiomyocytes.

**Figure 3:** mRNA and expression levels of ANP and BNP proteins in cardiomyocytes of each group.

**Figure 4:** Extracellular Ca^2+^ concentration of cardiomyocytes in groups.

**Figure 5:** CaN activities of calcineurin in cardiomyocytes of each group.

**Figure 6:** NFATc3 phosphorylation in the nucleus of cardiomyocytes of each group.

## Data Availability

The datasets used and/or analyzed during the present study are available from the corresponding author on reasonable request.
